# A Data-Driven Model for Automated Chinese Word Segmentation and POS Tagging

**DOI:** 10.1155/2022/7622392

**Published:** 2022-09-16

**Authors:** Qing Xu, Zhiyou Wang

**Affiliations:** ^1^Changsha University of Science and Technology, Changsha, Hunan 410000, China; ^2^School of Electronic Communication and Electrical Engineering, Changsha University, Changsha, Hunan 410000, China

## Abstract

Chinese natural language processing tasks often require the solution of Chinese word segmentation and POS tagging problems. Traditional Chinese word segmentation and POS tagging methods mainly use simple matching algorithms based on lexicons and rules. The simple matching or statistical analysis requires manual word segmentation followed by POS tagging, which leads to the inability to meet the practical requirements for label prediction accuracy. With the continuous development of deep learning technology, data-driven machine learning models provide new opportunities for automated Chinese word segmentation and POS tagging. Therefore, a data-driven automated Chinese word segmentation and POS tagging model is proposed in order to address the above problems. Firstly, the main idea and overall framework of the proposed automated model are outlined, and the tagging strategy and neural network language model used are described. Secondly, two main optimisations are made on the input side of the model: (1) the use of word2Vec for the representation of text features, thus representing the text as a distributed word vector; and (2) the use of an improved AlexNet for efficient encoding of long-range word, and the addition of an attention mechanism to the model. Finally, on the output side, an additional auxiliary loss function was designed to optimise the Chinese text based on its frequency. The experimental results show that the proposed model can significantly improve the accuracy and operational efficiency of Chinese word segmentation and POS tagging compared with other existing models, thus verifying its effectiveness and advancement.

## 1. Introduction

Over the past decades, natural language processing has received much attention in the field of machine learning, and its applications are widespread, such as data mining, system management, and opinion monitoring. With the rapid development of the contemporary information society and the increasing amount of textual information generated by the Internet, natural language processing techniques are becoming increasingly important. These vast amounts of data exist in different forms on the Internet and managing them using automated natural language processing methods is a daunting and commercially valuable task. Natural language is the language that humans need to use in their daily lives, studies, and work [1–5]. Natural language is a fundamental method of communication between people. Unlike artificially designed machine languages, natural languages are highly abstract, complex, and versatile. Natural language processing is the core technology that enables the exchange of information between humans and machines and is the backbone of artificial intelligence.

Currently, natural language processing techniques can be broadly divided into five levels [6–9]: phonological analysis, lexical analysis, syntactic analysis, semantic analysis, and pragmatic analysis. The purpose of lexical analysis is to determine the position, composition, and properties of words in a sentence according to syntactic rules. For Chinese natural language processing, lexical analysis mainly consists of two tasks: word segmentation and part-of-speech (POS) tagging [10–12]. Unlike phonetic writing, which is based on the Latin alphabet, Chinese is an ancient meaning-phonetic writing. Since there are no natural spaces between words in a sentence, word segmentation is a unique and important part of natural language processing in Chinese. POS tagging requires that each word be given a lexical label. POS is the most basic grammatical feature of words, indicating their composition and role in a sentence [13, 14]. Word segmentation and POS tagging are the most fundamental techniques in natural language processing, apart from speech analysis. Word segmentation and POS tagging have a crucial impact on upper-level tasks such as syntactic analysis, text classification, and machine translation.

On the other hand, deep learning, a branch of machine learning, has once again seen a surge in research as the amount of data has exploded and computing power has increased [15–18]. Compared with traditional statistical-based machine learning, data-driven deep learning no longer requires researchers to spend too much time and effort on feature engineering. Data-driven deep learning can automatically learn and extract features from large amounts of data; thus, unlocking the potential value of large amounts of data [19–22]. In view of the great success of deep learning in the field of computer vision, many researchers have started to try to use deep learning techniques to solve natural language processing problems and have gradually accumulated a lot of research experiences and application results. As the underlying core technology of Chinese natural language processing, the study of Chinese word segmentation and POS tagging has great theoretical and practical significance. However, deep learning has not achieved significant advantages over traditional statistical analysis methods in the area of Chinese word segmentation and POS tagging, suggesting that there is still room for further research and optimisation of the problem.

Therefore, the purpose of this research is to apply the data-driven deep learning technology to Chinese word segmentation and part-of-speech tagging tasks, so as to achieve the automation of these two tasks at the same time with high precision.

The rest of the paper is organised as follows: related works are presented in Section 2. In Section 3, the proposed data-driven automation-based model was studied in detail, while Section 4 provides the optimisation of the input layer. The optimisation of the output layer is presented in Section 5, while Section 6 provides the experimental results and analysis. Finally, the paper is concluded in Section 7.

## 2. Related Work

Research on Chinese word segmentation began in the 1990s. The earliest Chinese word segmentation methods were lexicon- and rule-based methods, such as forward maximal matching, reverse maximal matching, and least word cut. Although lexicon- and rule-based methods were easier to implement, the accuracy of word segmentation was low. Hong et al. [23] proposed to use the Google News corpus to handle lexicon-based Chinese word segmentation tasks. Chang et al. [24] introduced conditional random fields into Chinese word segmentation, which has become the mainstream method for Chinese word segmentation. Most of the word segmentation methods based on word-related feature learning use semiconditional random fields, and thus need to assign the same label to multiple consecutive words in each step, resulting in long training time.

POS tagging refers to assigning each word in a sentence a category called part-of-speech. POS is the most basic grammatical property of a vocabulary. Accurate POS tagging will bring great advantages to upper-level tasks such as syntactic analysis. The earliest approaches to POS tagging were rule-based methods. Although rule-based approaches have a relatively simple theory, they require a lot of time to manually write various complex rules. Wang et al. [25] proposed an error-driven machine learning method that automatically learns lexical transformation rules; thus, reducing the workload of writing rules manually to a certain extent. With the development of statistical machine learning, POS tagging was modelled as a sequence tagging problem. The algorithms that can be used for the sequence tagging problem can basically be used to solve the POS tagging problem, such as support vector machines, hidden Markov models, maximum entropy models, and conditional random fields. Tursun et al. [26] used hidden Markov models for English POS tagging and achieved 95% tagging accuracy.

With the rise of deep learning, deep neural network-based POS tagging methods have also received much research. Liu et al. [27] first proposed a neural network-based Chinese word segmentation method in 2019, verifying the feasibility of deep learning on the Chinese word segmentation task. Su et al. [28] proposed a recurrent neural network with gate structure and used it to extract n-gram features in the Chinese word segmentation task. Deep learning-based Chinese word segmentation methods have been the mainstream approach in the field of Chinese word segmentation research in recent years, and many successful experiences have been achieved. However, there is still room for improvement in the accuracy and training efficiency of deep learning-based word segmentation methods compared to traditional word segmentation methods.

AlexNet is the first deep convolutional neural network model for image classification [29–34] and is a historically important model in the field of convolutional neural networks. Therefore, this paper uses the AlexNet model to simultaneously perform Chinese word segmentation and POS tagging in one complete step. In order to improve the model accuracy and operational efficiency, the input and output of the model are optimised in this paper.

The main innovations and contributions of this paper include the following:

1. The AlexNet network was improved in the input to the model to reduce the number of model parameters, resulting in a faster training and learning speed. In addition, an attention mechanism was added to the AlexNet network to efficiently learn the contextual semantics of the target words. Word weights are adjusted during the training process based on the relevance of the input to the word vector to the final predicted outcome.
2. Additional auxiliary loss functions were designed to optimise the output of the model based on the Chinese text frequencies.

## 3. Data-Driven Automation-Based Model

In the field of Chinese natural language processing, word segmentation and POS tagging are regarded as two separate processing steps. In other words, for a Chinese sentence, a word segmentation model is used to segment the words, and then a POS tagging model is used to annotate the lexical properties of the segmented words. This approach is also known as the pipeline model. In this model, word segmentation and POS tagging are two steps, one after the other, and the POS tagging depends on the outcome of the segmentation while the segmentation is not affected by the POS tagging in any way. This pipeline model has two obvious drawbacks: the problem of error transmission and word segmentation cannot sense POS information. The former refers to the fact that errors in word segmentation are passed on to POS tagging. The latter refers to the fact that the POS information is not directly considered in the segmented model itself. To address these two issues, this paper decides to use a joint model that is entirely word-based. This paper argued that word segmentation has a large impact on POS tagging and that they should not be considered as two separate processing steps. Therefore, this paper attempts to reduce the error rate of POS tagging by using only one model to deal with both Chinese word segmentation and POS tagging at one time.

### 3.1. Overall Model Architecture Design

The overall architecture of the joint model proposed in this paper is shown in Figure 1.

Firstly, the input layer needs to represent each word as a vector. This is because the model in this paper is entirely word-based and therefore word vectors must be used as the basic input to the network. In this paper, text word features are extracted using word2Vec so that the text is represented as a distributed word vector. Considering the complex combinatorial relationships of Chinese words, an AlexNet network model is also used for further feature extraction of the word vectors after the input of the distributed word vectors.

The hidden layer refers to the intermediate layer in a broad sense, rather than the hidden layer in a general feed-forward neural network. In order to make full use of the syntactic and semantic information contained in the original corpus, this paper introduces a neural network language model as a secondary task to be trained jointly with the main task. The output layer predicts a label for each word in the sentence. In order to explicitly model the dependencies between tags, the classical conditional random field is used in the output layer for tag prediction. At the same time, an auxiliary loss function is added to the output side of the model for predicting the word frequencies at the corresponding positions; thus, improving the training effect of the whole model.

### 3.2. Labeling Strategy

The Chinese word segmentation tags indicate the relative position of a character in a word, as shown in Table 1, and mainly include binary tag sets, ternary tag sets, and quaternary tag sets. The greater the number of tags, the greater the number of positions that can be represented, but at the same time the complexity of the model increases and the efficiency of both training and prediction decreases. Conversely, the smaller the number of tags, the more efficient the model, but the less accurate it is. Considering the accuracy and efficiency of the model, this paper uses a quaternary tags set (*B*, *I*, *E,* and *S*) to represent the boundaries of a word [35]. *B* means the current character is the first character of the word, *M* means the current character is in the middle of the word, *E* means the current character is the last character of the word, and *S* means the current character is a single word.

### 3.3. Neural Network Language Models

Current supervised sequence tagging methods based on manually annotated corpora tend to make use of the tagging information alone, without making use of the information in the original corpus itself. The size of the manually annotated corpus is very limited due to cost and financial constraints; in contrast, the size of the unannotated raw text is getting larger and larger. Therefore, how to make full use of the unannotated original text becomes the key issue to be considered in this paper. Word vector-based methods such as word2vec are a shallow approach. The models are not able to capture the high-level information of natural language in the pretraining process of word vectors by using word2vec techniques alone. Neural network language models can effectively solve this problem, as shown in Figure 2.

Pretrained word vectors based on large-scale raw text are an effective way to extract information from the original paper, and the resulting word vectors have some ability to characterise the semantics. However, as the lowest-level input to the model, the pretrained word vector itself is only a shallow feature representation and lacks richer high-level information. Therefore, this paper proposes the use of neural network language models as an alternative method of extracting information from raw text.

(1) $$\begin{array}{c} P_{f}\left(c_{1},\cdots ,c_{n}\right)=\overset{N}{\underset{i=1}{\prod }}P_{f}\left(\left.c_{i}\right|c_{1},\cdots ,c_{i-1}\right)\text{,} \end{array}$$

where *c*_*i*_ indicates the character to be predicted at the current moment and *c*_1_, ⋯, *c*_*i*−1_ indicates all the characters in the text.

(2) $$\begin{array}{c} P_{f}\left(\left.c_{i}\right|c_{1},\cdots ,c_{i-1}\right)=\frac{\exp\;\left(w_{c_{i}}^{T}f_{i-1}\right)}{\underset{{\hat{c}}_{j}}{\sum }\exp\left(w_{{\hat{c}}_{j}}^{T}f_{i-1}\right)}\text{,} \end{array}$$

where *w*_*C*_*i*__ represents the weight vector corresponding to*c*_*i*_ and *f*_*i*−1_ represents the output of the neuron. Thus, the training objective function of neural network can be obtained.

(3) $$\begin{array}{c} F=-\frac{1}{N}\underset{i}{\sum }\log P_{f}\left(c_{i}\right)\text{.} \end{array}$$

### 3.4. Conditions Follow the Airport

In the input layer, for each word of a sentence, there is a corresponding word vector. After a hidden layer consisting mainly of a neural network language model, we are given a corresponding output vector. The output vector models the contextual information of the sentence adequately. The next step is to predict the final output labels based on the output vector. There are obvious dependencies between the output labels, so it is often necessary to explicitly model the label dependencies at the output layer. Conditional random fields (CRFs) [36–38] are suitable for exactly this need. A CRF is a model of conditional probability distribution. By manually designing suitable feature templates, conditional random fields can obtain a strong feature fitting capability, resulting in a large number of feature functions. Conceptually, CRF is a probabilistic undirected graph model.

For the input sentence*x*=(*c*_1_, ⋯, *c*_*n*_), the corresponding sequence of output labels is *y*(*z*)=(*y*_1_, ⋯, *y*_*n*_). Given *z*, a CRF probability model can express the conditional probability of *y*.

(4) $$\begin{array}{c} p\left(\left.y\right|z;W,b\right)=\frac{\overset{n}{\underset{i=1}{\prod }}\psi_{i}\left(y_{i-1},y_{i},z\right)}{\underset{y^{\prime }\in Y\left(z\right)}{\sum }\overset{n}{\underset{i=1}{\prod }}\psi_{i}\left({y^{\prime }}_{i-1},{y^{\prime }}_{i},z\right)}\text{,} \end{array}$$

where *ψ*_*i*_(*y*_*i*−1_, *y*_*i*_, *z*) denotes the potential energy function in the CRF. *W* and *b* denote the weight vector and bias vector corresponding to the label(*y*′, *y*), respectively. In the training phase, maximum likelihood estimation is used with the objective of maximising the conditional likelihood.

(5) $$\begin{array}{c} J_{CRF}=-\underset{i}{\sum }\log p\left(\left.y_{i}\right|z_{i}\right)\text{.} \end{array}$$

In the test or decoding phase, the objective is to search for the globally optimal sequence of labels *y*^*∗*^, that is, to require the maximum conditional probability.

(6) $$\begin{array}{c} y^{*}=\underset{y\in Y\left(z\right)}{argmax}p\left(\left.y\right|z;W,b\right)\text{.} \end{array}$$

## 4. Optimisation of the Input Layer

### 4.1. Word Vector Representation of Text

The distributed representation of the word vector word2Vec [39] mainly consists of CBOW and skip-gram, where the structure of CBOW is very similar to that of a neural network language model, as shown in Figure 3. CBOW uses a strategy where all words share a hidden layer to achieve efficient model training. The input to CBOW is contextual and requires vector summation. Skip-gram predicts context based on the central word. Skip-gram can be represented as maximising the log conditional probability.

The CBOW model consists of three layers: input, projection, and output. For the word sequence(*𝒲*_*t*−2_, *𝒲*_*t*−1_, *𝒲*_*t*_, *𝒲*_*t*+1_, *𝒲*_*t*+2_), *w*_*t*_ is the current word and the rest of the words are their contexts. The projection layer is used for the accumulation of input layers, thus obtaining *X*_*w*_. Random negative sampling is performed in the output layer to achieve the prediction. Assuming that the given context *wis* a positive sample and the other words are negative samples, any word *v* can be represented as follows:

(7) $$\begin{array}{c} L^{w}\left(v\right)=\left\{\begin{array}{c} 1,v=w\\ 0,v\neq w \end{array}\right.\text{,} \end{array}$$

where *L*^*w*^(*v*) denotes the label of word *v*. 1 represents a positive sample, and 0 represents a negative sample. For a given positive sample (Context(*w*)*w*), the final goal is to maximize *G*.

(8) $$\begin{array}{c} G=\log_{2}\prod_{w\in C}g\left(w\right)\text{,}\\ g\left(w\right)=\prod_{u}p\left(\left.u\right|Context\left(w\right)\right)\text{.} \end{array}$$

In general, if the probability of a negative sample decreases, the probability of a positive sample increases. Given the context, CBOW will derive the target words. In this paper, the CBOW model will be used to train the word vectors. Word2vec word vector training parameters are shown in Table 2.

In addition, as the traditional word vector would ignore the order of words and their relationships in the text, the training time will be too long. Therefore, this paper modifies the text representation model on the basis of the traditional word representation, as shown in Figure 4. Topic categories between different texts are trained using LDA estimation. The topic categories are combined with the top-ranked words to generate a hybrid representation model. Related studies have shown that this hybrid representation can improve prediction accuracy and reduce training time. In addition, this hybrid representation is suitable for unbalanced data classification.

### 4.2. Improved AlexNet Based on Attention Mechanism

First, word2Vec was used to word represent the text and train word vectors; thus, representing natural language in the form of distributed vectors. Then, a one-dimensional convolution was used in the convolutional layer, which aimed to reduce the number of text encoding features. Next, a modified AlexNet was used to efficiently encode long-range words. Finally, the text feature representations are fed into the attention layer, which selects features that are highly relevant to the final classification result as the final output.

AlexNet is a derivative model of CNN. However, the training time for AlexNet is long; therefore, this paper makes further improvements to the AlexNet network. The improved AlexNet replaces the location of the fully connected layer with a convolutional layer and removes the LRN layer.  Figure 5 shows the structure of the improved AlexNet, which is divided into 8 layers: layers 1 to 5 are convolutional layers, while layers 6 to 8 are fully connected layers. The activation function is a ReLU function, which acts as a nonsaturating nonlinear function to speed up the convergence of the model. Dropout layers are added after layer 6 to prevent overfitting problems. The final layer has no activation function. The improved AlexNet inherits many of the features of AlexNet, such as easier parallelisation operations.

The role of the convolutional layer is to extract the semantics of the text. It is generally possible to preserve the convolutional layers and pretrained parameters during the extraction process from shallow semantics to advanced semantics. In this paper, the first five conv layers of AlexNet are preserved and some FC layers are removed. The parameters of the improved AlexNet are shown in Table 3. The improved AlexNet can quickly extract the underlying semantic features from the original text and reduce the number of dimensions.

Attentional mechanisms were first used to model the attentional behaviour of the human brain [40, 41]. In the improved AlexNet, the conv layer narrows down the input features used in prediction. However, for all input words, the correlation between each word and the final prediction is not the same. The use of a one-dimensional convolutional layer reduces the number of features needed to encode text.

The improved AlexNet in this paper receives the features generated in the conv layer stage and generates them by extracting the last hidden layer. The improved AlexNet is able to access contextual information and treats the obtained information as two different text representations. The text features are fed into the improved AlexNet model, which generates a feature representation of the sequence. This feature representation is then fed into the attention layer, which selects the features that are highly relevant to the final classification result. Using such processing, the attention mechanism can efficiently learn the contextual information surrounding the target word, thereby significantly improving prediction accuracy and reducing the number of weights required for prediction.

Bahdanau attention model is used in attention mechanism. Based on the hidden vector of word vectors*h*_*j*_ and the weights *α*_*ij*_, the vector of contextual words for the *i-*th target word *c*_*i*_ can be calculated.

(9) $$\begin{array}{c} c_{i}=\overset{T}{\underset{j=1}{\sum }}\alpha_{ij}h_{j}\text{.} \end{array}$$

The formula for calculating the weights is shown as follows:

(10) $$\begin{array}{c} \alpha_{ij}=\frac{\exp\left(e_{ij}\right)}{\overset{T}{\underset{k=1}{\sum }}\exp\left(e_{ik}\right)}\text{.} \end{array}$$

### 4.3. Loss Functions

The improved AlexNet model was trained using a minimized cross-entropy loss function so as to fit a linear softmax classifier.

(11) $$\begin{array}{c} Loss\left(W\right)=-\underset{i\in Jt}{\sum }\underset{k}{\sum }y_{i,k}\ln\;\left(p\left(\left.y_{i,k}\right|v_{i};W\right)\right)\text{,} \end{array}$$

where *W* denotes *the* network model weights and v_*i*_ (*i* ∈ {1,..., n}) denotes the attribute of the *i-*th text.

## 5. Optimisation of the Output Layer

Looking at the word segmentation results, it was found that there were a very high number of occurrences of common words in the training corpus. The model was sufficiently trained on the frequently used words, so the tagging results were more accurate. However, due to the relatively small number of occurrences of rare words, the model is not sufficiently trained on rare words, resulting in poor tagging results, which can be regarded as a kind of “Hard Examples”. This small number of hard examples can lead to a decrease in the overall performance of the model. If we can improve the accuracy of the tagging of the rare characters, the overall performance of the model will also be improved. It was found that the frequency of Chinese characters approximately conforms to Ziff's law. This empirical law has been validated in many fields and is also known broadly as the two-eight law.

A small number of high-frequency words appear very often, and a large number of low-frequency words appear very rarely. The low-frequency characters are therefore the “Hard Examples” of the task. Considering the characteristics of this character frequency distribution and not wanting the model to be too complex, this paper proposes a simple approach to solve this problem. An auxiliary loss function is added to the output side of the model to predict the word frequencies at the corresponding positions. This loss function is intended to aid the training of the whole model and is expressed as a squared difference loss function.

(12) $$\begin{array}{c} J_{{\text{char }}_{-}\text{freq }}=\underset{i}{\sum }{\left(f_{i}-{\hat{f}}_{i}\right)}^{2}\text{,} \end{array}$$

where *f*_*i*_ indicates the predicted word frequency of the *i-th character* in the sentence and $\hat{f}$ indicates the true word frequency of the *i-th* character.

By adding the auxiliary loss function described above, the model is explicitly guided to predict word frequencies. The auxiliary loss function gives the model the ability to distinguish between high- and low-frequency words, which improves the accuracy of the model for low-frequency words. The experiments show that the auxiliary loss function does have a positive effect on the tagging results.

## 6. Experimental Results and Analysis

### 6.1. Experimental Parameter Settings

In this paper, a data-driven automated Chinese word segmentation and POS tagging model is implemented using the Python programming language and Google's TensorFlow deep learning framework. The key parameters of the automated model are shown in Table 4. The model is trained using gradient descent-based backpropagation, where the batch size is set to 32 and the maximum number of training sessions is 30. The number of convolutional layers used for word feature extraction is set to 3.

The larger the dimension of the word vector, the better the model training results. However, when the dimension of the word vector is large enough, the increase in the dimension of the word vector is very small. However, the larger the word vector dimension is, the slower the model can be trained and tested. Therefore, we choose to set the word vector dimension to 64 to find a good compromise between model effectiveness and speed.

Dropout is an extremely common technique in the field of deep learning and is very important in mitigating model overfitting; Dropout is to some extent similar to L2 regularisation; the core idea of Dropout is to drop a number of neurons at random with a certain probability during model training, so that the weights of the neurons can represent various aspects of the input data, rather than concentrating on certain elements. This method introduces random noise, which can be used to create a new model. This method of introducing random noise can increase the sparsity of the network and has the effect of alleviating model overfitting. Experiments in this paper found that dropping neurons at random with a 20% probability worked best.

### 6.2. Experimental Data and Evaluation Indicators

Three different publicly available datasets were used to test the proposed automated model, as shown in Table 5. Ninety percent of each dataset was randomly selected as the training set, while the remaining 10% was used as the test set.

This paper evaluates the performance of the automation model using the micro-*F*1 metric (micro-*F*1) and the macro-*F*1 metric (macro-*F*1). Higher values of micro-*F*1 and macro-*F*1 indicate stronger performance.

(13) $$\begin{array}{c} \text{Micro}\_F1=\frac{2\times p_{t}\times r_{t}}{p_{t}+r_{t}}\text{,} \end{array}$$

where *p*_*t*_ indicates the total accuracy and *r*_*t*_ indicates the total recall.

(14) $$\begin{array}{c} {Macro}_{F1}=\frac{2\times p_{m}\times r_{m}}{p_{m}+r_{m}}\text{,} \end{array}$$

where *p*_*m*_ represents the mean of accuracy and *r*_*m*_ represents the mean of recall.

### 6.3. Performance Comparison

The proposed automated model was compared with Bi-LSTM [42], CNN [43], and BiRNN [44] on the above three publicly available datasets, and the experimental results are shown in Figure 6. It can be seen that the performance of the method in this paper on two datasets (MSR and CTB7) is significantly better than the other methods. On the CTB5 dataset, the BiRNN method is closer to the method in this paper. Overall, this method achieves better text classification performance. This is mainly due to the fact that the proposed method adds an attention mechanism to the AlexNet-2 architecture, which adjusts the weights according to the relevance of each input to the final prediction result.

A comparison of the average time required for the training of the four models is shown in Figure 7. It can be seen that the proposed automated model is slightly faster than the Bi-LSTM model. Although both models use an attention mechanism, the improved AlexNet framework has fewer parameters and a lighter structure. The two models, CNN and BiRNN, take more time to tune the parameters, resulting in longer running times.

## 7. Conclusion

In order to implement automated Chinese word segmentation and POS tagging, this paper proposes a data-driven automation model. The proposed model consists of three parts: an input layer, a hidden layer, and an output layer. The input layer uses word2Vec to extract textual word features, and a modified AlexNet network model is used to further extract features from the word vectors. The hidden layer introduces a neural network language model as a secondary task for joint training with the main task. The classical conditional random field was used in the output layer for label prediction. At the same time, an auxiliary loss function is added to the output side of the model for predicting the word frequency at the corresponding position; thus, enhancing the training effect of the whole model. The experimental results show that the proposed model has a certain improvement in both micro-*F*1 metrics and macro-*F*1 metrics compared with other models and also has a high operational efficiency.

## Figures and Tables

**Figure 1:** Joint model architecture.

**Figure 2:** Architecture of neural network language model.

**Figure 3:** CBOW neural network model.

**Figure 4:** Hybrid representation.

**Figure 5:** Structure of the improved AlexNet.

**Figure 6:** Accuracy comparison results: (a) MSR data set, (b) CTB7 dataset, and (c) CTB5 dataset.

**Figure 7:** Comparison of the average time spent in training.

**Table 1:** Examples of Chinese word segmentation tag sets.

	Tag	Description
Quaternary tag set	*B*	Beginning
	*M*	Middle
	*E*	Ending
	*S*	One-character words
Ternary tag set	*B*	Beginning
	*I*	Middle or end
	*0*	One-character words
Binary tag set	*B*	Beginning
	*NB*	Not the beginning

**Table 2:** Word2vec word vector training parameters.

Parameter name	Meaning of parameter	Parameter value
Alpha	Initial learning rate	0.01
Size	Vector dimension	64
Mincount	Minimum word frequency	5
Window	Context window size	15
Negative	Number of negative samples	20

**Table 3:** Parameters of the improved AlexNet.

Layer	Convolution kernel size	Step length	Number of cores
Convolutional layer 1	11 × 11 × 3	4	96
Pooling layer 1	1 × 3 × 3 × 1	2	—
Convolutional layer 2	5 × 5 × 48	1	256
Pooling layer 2	1 × 3 × 3 × 1	2	—
Convolution layer 3	3 × 3 × 384	1	256
Convolutional layer 4	3 × 64 × 384	1	384
Convolutional layer 5	3 × 3 × 256	1	384
Pooling layer 5	1 × 3 × 3 × 1	2	—
Fully connected layer 6	32 × 256	—	256
ReLU6	—	—	384
Dropout layer	—	—	—
Fully connected layer 7	32 × 256	—	256
ReLU7	—	—	256
Dropout layer	—	—	—
Fully connected layer 8	256 × 2	—	2
Prob	Softmax	—	—
Output	—	—	—

**Table 4:** Key parameters of the automation model.

Parameter	Numerical value
Number of AlexNet hidden layer nodes	200
AlexNet network depth	2
Number of AlexNet convolutional layers (pooling layers)	3
Dropout	0.2
Training optimiser	AdaGrad
Initial learning rate	0.1
Batch size	32
Word vector dimension	64

**Table 5:** Presentation of the four datasets.

Dataset	Data segmentation	Number of words (K)	Number of sentences (K)
MSR	Training set	494	18
	Test set	8.0	348
CTB7	Training set	78	31
	Test set	245	10
CTB5	Training set	2131	78
	Test set	107	4

## Data Availability

The experimental data used to support the findings of this study are available from the corresponding author upon request.
